# Predictors of Smoking Preventive Behavior Based on Empowerment Components among Male Students of High Schools: A Cross-Sectional Study in Iran

**DOI:** 10.1155/2023/4223794

**Published:** 2023-01-31

**Authors:** Alireza Didarloo, Naser Sharafkhani, Baratali Rezapour, Fatemeh Moghaddam-Tabrizi

**Affiliations:** ^1^Social Determinants of Health Research Center, Clinical Research Institute, Urmia University of Medical Sciences, Urmia, Iran; ^2^Faculty of Health, Isfahan University of Medical Sciences, Isfahan, Iran; ^3^Department of Public Health, Faculty of Health, Urmia University of Medical Sciences, Urmia, Iran; ^4^Reproductive Health Research Center, Urmia University of Medical Sciences, Urmia, Iran

## Abstract

**Background:**

Smoking among adolescents and young adults is believed to be one of the most important preventable health problems. The etiology of smoking is one of the most pivotal activities in designing prevention programs. The aim of this study was to determine the correlates between components of empowerment in the context of smoking prevention in adolescents.

**Methods:**

This cross-sectional descriptive study was carried out on 422 high school male students in spring 2020. The data collection tool of this study was a valid and reliable researcher-made questionnaire containing demographic characteristics, items related to various components of empowerment, and items related to the smoking preventive behavior (SPB). A linear regression model was used, where the “SPB” outcome variable assumed three possible values: sensation seeking, problem-solving skills, self-efficacy, self-esteem, dependence on group, and attitude towards smoking reported in the previous literature were taken as independent variables, and smoking preventive behavior was considered as a dependent variable.

**Results:**

The results revealed that 10.42% of the students were active smokers and 40.75% of them had the experience of smoking. The results also showed a positive and significant relationship between problem-solving skills (*r* = 0.394, *P* < 0.001), self-efficacy (*r* = 0.340, *P* < 0.001), self-esteem (*r* = 0.310, *P* < 0.001), and attitude (*r* = 0.333, *P* < 0.001) with the SPB. In addition, a negative and significant correlation was observed between group dependence (*r* = -0.313, *P* < 0.001) and the SPB. Overall, the components of empowerment were able to explain 26.5% of the variance in the SPB. Among the components, problem-solving skills solely explained 15.5% of variance of the SPB.

**Conclusion:**

According to the results of this study, it can be said that most adolescents are at risk of smoking. Explanatory factors for adopting the SPB include improving problem-solving skills, creating a negative attitude towards smoking, increasing self-efficacy to prevent smoking, reducing group dependence, and increasing self-esteem in adolescents. Multilevel interventions and actions by policymakers, educators, and related organizations to prevent adolescent smoking and educate them about adolescent empowerment skills to prevent smoking should be considered.

## 1. Background

Smoking is a high-risk human behavior that imposes great economic and social costs on communities [1]. An extensive use of tobacco is known as a health and epidemic problem in adolescents [2].

The World Health Organization (WHO) has estimated that 8 million people die annually from tobacco-related diseases by 2020 [3]. The WHO emphasizes that if the current trend of smoking continues, by 2030 the number of victims will be 10 million [4], 70% of which will occur worldwide in developing countries [5].

Smoking causes 90% of lung cancers, 40% of other cancers, 75% of respiratory diseases, 50% of cardiovascular diseases, and 12% of all deaths. [6] More than $ 150 billion is spent annually on health problems caused by smoking [7]. Despite the fact that the harms of smoking have been well established, many adolescents are still interested in smoking [8, 9]. The age of onset of smoking has decreased in developed and developing countries [10], and approximately 90% of smokers experienced smoking at younger ages [11]. The lower the age of onset of smoking, the more dependent the smoker on this habit, which would ultimately lead to prolonged smoking [12].

The prevalence of smoking in different parts of the world varies from 14.2% to 39% [13, 14]. In Iran, the prevalence of smoking is 9.2% to 28.8%, which has been estimated to be 14.2% in adolescents [15]. Adolescence is a critical period of development since during this period, many positive health behaviors (such as diet and exercise) and dangerous health behaviors (such as smoking and alcohol consumption) are formed. [16] One of the most important requirements for a country to achieve economic, social, and political progress and stability is to pay attention to the health and developmental needs of this age group [17].

One of the concerns of health/social policymakers in today's society is the increasing prevalence of addictive behaviors, especially smoking addiction in adolescents [18–20].

Cigarette addiction treatment is expensive and difficult and requires a variety of treatment approaches, such as medication and psychotherapy. However, even the most effective treatments are associated with a high rate of recurrence of smoking, which is because susceptible environments, ease of access to cigarettes, social networks, and supporting smoking friends reduce the progress of smoking treatment and finally lead to its cessation [21].

Therefore, prevention of smoking is easier than addiction treatment and is considered as the most appropriate and logical solution [22]. Necessary requirements for the prevention of smoking include the analysis of smoking behavior among children, correcting misconceptions about smoking, empowerment of individuals against smoking since childhood, taking into account family pressures and crises of childhood, and the role of social variables [23, 24].

Empowerment is currently one of the most important concepts in community development [25]. The term empowerment was first used in texts of political and social sciences and soon found its place in management and health issues. [26] From the perspective of the WHO, empowerment, as the heart of health promotion [27], includes the process through which individuals gain further control over decisions and actions that affect their health [28].

Empowerment has different levels; empowerment at the individual level is the elimination of personal disabilities and the formation of a sense of personal power and self-efficacy. Interpersonal competence means having the ability to influence others [29].

To empower individuals, previous studies have emphasized improving components such as problem-solving skills, self-efficacy, self-control, self-esteem, emotional management, shifting attitude towards smoking, and adaptation towards environmental conditions [23, 30, 31]. In order to design appropriate prevention programs, it is necessary to be aware of the factors influencing the onset and persistence of smoking addiction. Over the recent years, one of the most important achievements in the field of theorizing and policymaking of prevention programs has been the emphasis on risky and protective factors as a descriptive and predictive framework [32].

Hence, this study was conducted to answer the key question of what are the correlates and the power of explaining various components of empowerment related to the prevention of smoking in children and adolescents? By answering this question, we can design and implement appropriate interventions and strategies to prevent smoking behavior in adolescents. We could also prevent and control the burden of diseases resulting from this problem.

## 2. Methods

This descriptive-analytical (cross-sectional) study was performed on 422 male students in high schools, spring 2020, in Urmia, Northwest Iran. In this study, to determine the sample size, preliminary data on smoking frequency were used in a pilot study that was performed on 100 students randomly. With the preliminary analysis on the data obtained from the pilot study and considering the minimum odds ratio about the relationship between the factors affecting cigarette consumption equal to 1.9 and with a confidence level of 95%, power of 80%, and considering the design effect of 1.5 and drop out Equivalent to 20% by using EPI INFO.2000 software to estimate the sample size, finally the sample size was estimated to be 420 people.

The study subjects were selected via multistage sampling method; primarily, Urmia city was divided into two central and peripheral districts. A list of secondary schools was then extracted from the Urmia Education Department. Twelve male schools were randomly selected from each district (a total of 24 high schools). Afterwards, in proportion to the number of students studying at different levels (1st, 2nd, and 3rd year) of education in these schools, the study samples (422 male students) were selected employing a simple random sampling method and entered the study. The inclusion criteria in this study were being 1st-, 2nd-, and 3rd-year male students and not having experienced mental and/or cognitive problems. All the subjects filled a written consent form to participate in the study. The exclusion criteria were filling the questionnaire incompletely. The youngest student was 15 years old, and the oldest one was 18 years old. Therefore, a written parental informed consent form, as well as written student assent, was obtained from all the participants in this study.

It should be noted that in the present study, the meaning of active smoking is “Students who have smoked 100 cigarettes in their lifetime and currently smoke cigarettes every day (daily) or some days (nondaily)”; the meaning of experienced smoking is “Students who have smoked at least 100 cigarettes in their lifetime, but say they currently do not smoke.”

### 2.1. Study Tools

The data collection tool of this study was a researcher-made questionnaire consisting of the following parts: Part 1 comprises demographic characteristics of the student and his smoking status. Part 2 includes items about different components of student empowerment, including sensation-seeking questions (with 10 items), for example, “ I don't like to experience any substance that has strange or dangerous effects”; problem-solving skills (with 10 items), for example, “when making decisions, I look at the consequences of all the ways and compare them to each other”; self-efficacy (with six items), for example, “I'm sure I can resist the temptation to smoke well”; self-esteem (with six items), for example, “I feel as though I have a lot of good attributes”; negative attitude towards smoking (with eight items), for example, “if a person consumes a small amount of cigarettes and drugs, he will definitely becomes addicted”; and belonging to the group (with seven items), for example, “I like to be noticed when I'm with others.” There were a total of 47 items based on the 5-point Likert scale, ranging from 5 (I strongly agree), 4 (I disagree), 3 (I have no idea), 2 (I disagree), to 1 (I completely disagree).

Part 3 includes items of the SPB (with six items), for instance, “when someone smokes next to me, I try not to be exposed to the smoke.” These items are rated on a 4-point Likert scale, ranging from 3 (always), 2 (often), 1 (rarely), to zero (not at all). The score of the subscales of the questionnaire was transformed linearly to a 0- to 100-point scale, with 100 indicating the best status and zero the worst. It should be noted that the main outcomes of the study are linearly transformed variables taken from the sum of the Likert-scale responses in Parts 2 and 3 of the questionnaire.

To determine the validity of the researcher-made questionnaire based on the study of valid sources [23, 30, 33, 34], the qualitative method of content validity was used (an experienced panel of experts, including health education specialists, psychologists, medicine, and preventive medicine). In this method, the experts are asked to examine the items of the questionnaires in terms of simplicity, clarity, relevance, and necessity and express their opinions and suggestions. After receiving the feedback and suggestions from the experts, the necessary amendments were made to the study tools. Finally, the validity of the tools was confirmed.

The reliability of the questionnaire was measured by Cronbach's alpha test method on 30 male students who were similar to the studied population in terms of demographic characteristics. The values were 0.71 for sensation seeking, 0.78 for problem-solving skill, 0.82 for self-efficacy, 0.79 for self-esteem, 0.74 for negative attitude towards smoking, 0.82 for group dependence, and 0.81 for the SPB, and ultimately, the instrument reliability was confirmed.

### 2.2. Data Analysis

The data collected in the SPSS software version 22 were analyzed using descriptive statistics, such as frequency and the mean and standard deviation. According to the results of the Kolmogorov–Smirnov test and the normality of data distribution, inferential statistics, such as Pearson's correlation coefficient test was used because regression analysis allows us to understand the strength of relationships between variables. Using statistical measurements such as R-squared/adjusted R-squared, regression analysis can tell us how much of the total variability in the data is explained by your model, and also, regression analysis tells us what predictors in a model are statistically significant and which are not; therefore, linear regression (stepwise) analysis (smoking preventive behavior was considered as a dependent variable, and problem-solving skills, negative attitude towards smoking, self-efficacy and self-esteem, sensation Seeking, and dependence on group were considered as independent variables) was used to analyze the data. In all the statistical analyses, the significance level was considered to be below 0.05.

## 3. Results

The response rate was 91.4% as 457 of 500 participants responded to the questionnaire, and 35(7%) questionnaires were incompletely answered, whereas incomplete questionnaires were excluded from the study.

In this study, 422 male students with an average age of 16.93 ± 0.76 were studied. The number of active smoking students was 44 (10.42%), and the number of those who experienced smoking was 172 (40.75).  Table 1 depicts an overview of the demographic characteristics of the samples.

The average score of the components related to students' empowerment associated with smoking prevention was not satisfactory. Based on the results of the study, the mean scores of the components of self-efficacy, self-esteem, sensation seeking, negative attitude towards smoking, group dependence, and problem-solving skills were 49.15 ± 7.68, 53.09 ± 6.98, 56.36 ± 5.25, 57.74 ± 5.83, 58.46 ± 6.98, and 59.57 ± 8.49, respectively (Table 2). In addition, the mean score of the SPB in the students was 55.56 ± 8.50 (Table 2).

The results of the Pearson correlation coefficient test showed that problem-solving skills, negative attitude towards smoking, self-efficacy, and self-esteem were positively and significantly related to the SPB. In addition, a significant and inverse relationship was observed between group dependence and the SPB, yet no significant relationships were found between the students' sensation seeking and the SPB (Table 3).

To determine the predictive power of empowerment components on the SPB, multiple linear regression analysis (stepwise method) was used. In this regression analysis, the components of problem-solving skills, self-efficacy, self-esteem, sensation seeking, group dependence, and negative attitude towards the SPB were entered in the regression equation. Based on the results, problem-solving skills, negative attitude towards smoking, group dependence, and self-efficacy were identified as the final predictors of the SPB in the students. In general, these variables were able to explain about 26.5% (*R*^2^ = 0.264) of the changes in the SPB (Table 4).

## 4. Discussion

In the study of any behavior, it is better to pay particular attention to the cause-and-effect relationships. The behavior of individuals could be attributed to different factors that need to be scientifically examined. The current work aimed to investigate the factors predicting the SPB based on different components of empowerment in students. According to the obtained results, 10.42% of the students were active smokers and 40.75% of them had a smoking experience.

Increasing the effectiveness of interventions in order to reduce smoking in adolescents necessitates the identification of the determinants of the SPB in this segment of population. Based on the results of the present study, there was a positive and significant relationship between problem-solving skills, negative attitude towards smoking, self-efficacy, and self-esteem with the SPB. Moreover, a significant and inverse relationship was observed between group dependence and the SPB, yet no significant relationships were found between the students' sensation seeking and the SPB. That is, those with problem-solving skills, self-efficacy, self-esteem, and a negative attitude towards smoking were more likely to engage in smoking preventive behaviors and those who felt more dependent on a group in which they participate were less likely to engage in the SPB.

In the present study, problem-solving skill was the strongest and most influential component of the behavior and was alone able to predict 15.5% of the changes in the SPB in the students. Problem-solving skill is a kind of goal-oriented thinking, [35] a mental process, and logical and systematic thinking, which helps a person to find multiple solutions once dealing with problems, such as addiction and smoking, and then find the best solution. [36].

The study of Parsian et al. revealed that adolescent problem-solving skills are a major predictor in the prevention of addiction and smoking. Their results are consistent with those of the present study. [37] Hitchcock also points out that one of the key points in the discussion of substance abuse, such as smoking, is paying attention to skills, such as problem-solving skills, which enable people to deal with problems. [38].

Negative attitude towards smoking are the second component of empowerment, which explained the SPB in students. The study of Morvati Sharifabad et al. revealed that creating negative attitude towards smoking in adolescents through various educational programs regarding the individual and social effects of this dangerous behavior could be effective on adolescents' reluctance to smoking. [39] Various studies have shown that teenagers believe that smoking is a way to gain social status and comfort. This unhealthy behavior should be controlled by reducing their positive attitude towards smoking and creating a negative attitude towards it [40, 41].

Self-efficacy was the third component of empowerment predicting the SPB in students. Bandra considers self-efficacy to be the most important prerequisite for behavior change and predictor of behavior. [42] In the study of Panahi et al., self-efficacy was mentioned as an important component in predicting the behaviors that prevent smoking. [33] According to Ghasemi et al., nonsmoking students had a high ability not to consume, whereas consumer students had a low ability to quit smoking due to certain problems, such as peer pressure or loss of fun with friends. [43] On the one hand, this could be due to the connection and friendship with peers who consume tobacco, and on the other hand, belonging to a group is one of the important needs of adolescents. [44] Given the importance of self-efficacy in performing healthy behaviors, increasing the life skills of students, particularly the skill of saying no and their resistance to peer pressure, could be considered for improving their self-efficacy.

According to the obtained findings herein, the feeling of belonging to a group was found to be the fourth component associated with students' empowerment concerning smoking preventive behavior. Learning any behavior occurs more profoundly from the groups that are closer to an individual; thus, these groups also act as outstanding role models for the individual. [45] In general, if the group to which a person belongs is involved in deviant actions, in fact the individual considers that group as a role model. [46] Hawkins' model of social development explains abnormal behaviors, including substance use (smoking and other addictive substances), based on social bonding. This model points to three effective factors in reducing a person's commitment to society, namely the pressures of a huge difference between goals and the individual's perception of the availability of the necessary conditions to achieve those goals, social disorder, and the process of socialization. According to this theory, emotional attachment to groups and peers who use addictive substances is considered to be the leading cause of substance abuse. [47] For note, it is not that a single factor is a necessary and sufficient condition for substance abuse (smoking), but that the substance abuse is a combined result of various factors. Some of these factors increase the risk of consumption, and others prevent and reduce drug use.

However, this study, like other studies, had its limitations. To begin with, this study is a cross-sectional study and cannot be used to examine the cause-and-effect relationship. Accordingly, it could be recommended that stronger studies be used for this purpose. Furthermore, the obtained results could not be generalized beyond the study sample and can be therefore generalized only to populations with similar features. Finally, the data collection tool in this study was a self-report questionnaire and the participants may have underestimated or overestimated their smoking preventive behavior, which may have affected the outcomes.

## 5. Conclusion

Based on the results of this study, the empowerment components predicted 26.5% of the variance in smoking preventive behaviors in students. Problem-solving skills, negative attitude towards smoking, self-efficacy, and dependence on group were the strongest predictors of smoking preventive behaviors, respectively, and these above-mentioned empowerment components to prevent smoking in adolescents were estimated at a low level, which requires measures and programs to improve these components. The obtained findings of the present study could be conducive to the development of ecological health promotion strategies, including family, school, and community organizations, such as youth affairs organization, municipality, and education. Implementation of cigarette use prevention and intervention programs for adolescents is warranted, and research on the effectiveness of such initiatives is necessary.

## Figures and Tables

**Table 1:** Characteristics of the study participants.

		Statistical index	
Variable		Mean (N)	SD (%)
Age		16.93	0.76

Grade	First grade of high school	155	36.7
	Second grade of high school	164	38.9
	Third grade of high school	103	24.4

Smoking status in students	Students who were active smokers	44	10.42
	Students who have experienced smoking	172	40.75
	Students were nonsmokers	206	48.82

**Table 2:** Mean scores of the various components of empowerment and the SPB in students.

	Statistical index			
Variable	Mean	Standard deviation	Maximum	Minimum
Sensation seeking	56.36	5.25	80	38
Problem-solving skills	59.57	8.49	78	34
Self-efficacy	54.81	7.68	75.2	33.3
Self-esteem	61.22	6.98	74.29	40
Dependence on group	58.46	6.12	77.14	34.2
Attitude towards smoking	57.01	6.98	72.5	40
Smoking preventive behavior	55.56	8.50	100	15.56

**Table 3:** Pearson's correlation coefficient of different components of empowerment with smoking preventive behavior in students.

Variable		Sensation seeking	Problem-solving skills	Self-efficacy	Self-esteem	Group dependence	Negative attitude towards smoking	Smoking preventive behavior
Smoking preventive behavior	r	0.082	0.394^*∗∗*^	0.340^*∗∗*^	0.310^*∗∗*^	−0.313^*∗∗*^	0.333^*∗∗*^	1
	p	0.091	0.001	0.001	0.001	0.001	0.001	

^*∗∗*^Correlation is significant at the 0.01 level (2-tailed).

**Table 4:** Steps of multivariate linear regression (stepwise) analysis in predicting smoking preventive behavior in students.

Criterion variable	Predictive variable	Correlation value (R)	Explanatory coefficient (R^2^)	Adjusted explanation coefficient
**Empowerment components**	Problem-solving skill	0.394	0.155	0.153
	Problem-solving skill and negative attitude towards smoking	0.474	0.225	0.221
	Problem-solving skill, negative attitude towards smoking, and self-efficacy	0.502	0.252	0.247
	Problem-solving skill, negative attitude towards smoking, self-efficacy, and group dependence	0.514	0.264	0.257

## Data Availability

The data used to support the findings of this study are available from the corresponding author upon request.

## Abbreviations

SPB: smoking preventive behavior
SPSS: Statistical Package for the Social Sciences
WHO: World Health Organization.

## References

[1] Who (2011). Economics of Tobacco Toolkit: Assessment of the Economic Costs of Smoking.

[2] Mathers M., Toumbourou J. W., Catalano R. F., Williams J., Patton G. C. (2006). Consequences of youth tobacco use: a review of prospective behavioural studies. *Addiction*.

[3] Rahnavard Z., Mohammadi M., Rajabi F., Zolfaghari M. (2011). An educational intervention using health belief model on smoking preventive behavior among female teenagers. *Journal of hayat*.

[4] Bollyky T. J. (2010). Beyond ratification: the future for US engagement on international tobacco control. *Center for Strategic and International Studies*.

[5] Petersen P. E. (2004). Continuous Improvement of Oral Health in the 21st century: The Approach of the WHO Global Oral Health Programme.

[6] Bartecchi C. E., MacKenzie T. D., Schrier R. W. (1994). The human costs of tobacco use. *New England Journal of Medicine*.

[7] Alexander W., Alexander L., Bader H., LaRosa J. (2013). *New Dimensions in Women’s Healthbook Alone*.

[8] Huang M., Hollis J., Polen M., Lapidus J., Austin D. (2005). Stages of smoking acquisition versus susceptibility as predictors of smoking initiation in adolescents in primary care. *Addictive Behaviors*.

[9] Abu Shomar R. T., Lubbad I. K., El Ansari W., Al-Khatib I. A., Alharazin H. J. (2014). Smoking, awareness of smoking-associated health risks, and knowledge of national tobacco legislation in Gaza, Palestine. *Central European Journal of Public Health*.

[10] Fleming C. B., Kim H., Harachi T. W., Catalano R. F. (2002). Family processes for children in early elementary school as predictors of smoking initiation. *Journal of Adolescent Health*.

[11] Ballard-Barbash R., Friedenreich C. M., Courneya K. S., Siddiqi S. M., McTiernan A., Alfano C. M. (2012). Physical activity, biomarkers, and disease outcomes in cancer survivors: a systematic review. *JNCI Journal of the National Cancer Institute*.

[12] Warren C. W., Lea V., Lee J., Jones N. R., Asma S., McKenna M. (2009). Change in tobacco use among 13-15 year olds between 1999 and 2008: findings from the Global Youth Tobacco Survey. *Global health promotion*.

[13] Deressa W., Azazh A. (2011). Substance use and its predictors among undergraduate medical students of Addis Ababa University in Ethiopia. *BMC Public Health*.

[14] El Mhamdi S., Wolfcarius-Khiari G., Mhalla S., Ben Salem K., Soltani S. (2011). Prevalence and predictors of smoking among adolescent schoolchildren in Monastir, Tunisia. *Eastern Mediterranean Health Journal*.

[15] Amin E. M., Rahimi M. A., Sahimi I. E., Hefazi M., Razaghi E. M., Yousefi N. R. (2007). The Prevalence of Smoking Among Iranian Middle School Students, a Systematic Review. *Iranian Journal of Psychiatry*.

[16] Williams P. G., Holmbeck G. N., Greenley R. N. (2002). Adolescent health psychology. *Journal of Consulting and Clinical Psychology*.

[17] Pettit G. S., Dodge K. A. (2003). Violent Children: Bridging Development, Intervention, and Public Policy. *Developmental Psychology*.

[18] Hammond S. K. (2009). Global patterns of nicotine and tobacco consumption. *Nicotine psychopharmacology*.

[19] Johnston L. D., O’Malley P. M., Bachman J. G., Schulenberg J. E. (2007). Monitoring the Future National Survey Results on Drug Use, 1975-2006. *Volume I: Secondary School Students*.

[20] Barrett A. E., Turner R. J. (2006). Family structure and substance use problems in adolescence and early adulthood: examining explanations for the relationship. *Addiction*.

[21] Maisto S. A., Connors G. J. (2006). Relapse in the addictive behaviors: integration and future directions. *Clinical Psychology Review*.

[22] Spoth R. L., Guyll M., Day S. X. (2002). Universal family-focused interventions in alcohol-use disorder prevention: cost-effectiveness and cost-benefit analyses of two interventions. *Journal of Studies on Alcohol*.

[23] Mohammadkhani S., Rezaei J. H. (2016). Relationship between Cigarette and Hookah Smoking with Individual, Family and Social Factors in Adolescents. *Journal of Sabzevar University of Medical Sciences*.

[24] Jazaery A., Rafiee H., Nazari M. (2003). The attitudes of middle school students in Tehran about addiction. *J University of social Welfare and rehabilitation science*.

[25] Khalili M. (2008). Pathology of the women’s participation in Iran’s contemporary society. *Women Studies*.

[26] Ghahremani M. G., Hasanzadeh M. (2015). The relative importance of organizational conditions in empowering managers. *International Journal of Organizational Leadership*.

[27] Haggart M., Carey P. (2000). *Community Health Promotion: Challenge for Practice*.

[28] Saffari M., Shojaeizadeh D., Ghofranipour F., Heydarnia A., Pakpour A. (2009). *Health Education & Promotion-Theories, Models & Methods*.

[29] Ehrhardt A. A., Sawires S., McGovern T., Peacock D., Weston M. (1999). Gender, empowerment, and health: what is it? How does it work? Journal of acquired immune deficiency syndromes. *JAIDS Journal of Acquired Immune Deficiency Syndromes*.

[30] Solhi M., Abasi H., Hazavehei M. M., Roshanaei G. (2014). Effect of educational intervention on empowerment of high school student in prevention of smoking. *Razi Journal of Medical Sciences*.

[31] Gordon J. R. (1993). *A Diagnostic Approach to Organizational Behavior*.

[32] Hawkins J. D., Catalano R. F., Arthur M. W. (2002). Promoting science-based prevention in communities. *Addictive Behaviors*.

[33] Panahi R., Ramezankhani A., Tavousi M., Osmani F., Niknami S. (2017). Predictors of Adoption of Smoking preventive behaviors among university students: application of health belief model. *Journal of Education and Community Health*.

[34] Habibi M., Besharat M.-A., Ferrer-Wreder L. (2012). A comp active study of smoking prevention indexes and effect of individual, family, and peers risk factors in adolescent’s smoking: smoker and non-smoker high school students. *Social Psychology Research*.

[35] Sarvghad S., Dianat A. (2009). A study of learning and problem-solving styles of University Students (A Case Study of Marvdasht Islamic Azad University). *Journal of New Approaches in Educational Administration*.

[36] Yuan H. B., Williams B. A., Fang J. B., Pang D. (2012). *WITHDRAWN: The Relationship between Self-Directed Learning Readiness and Problem Solving in Chinese Baccalaureate Nursing Students*.

[37] Parsian M., Hashemian K., Abolmaali K., Mirhashemi M. (2015). Prediction of drug attitude in adolescents based on family training risk factors for mental health in society: designing a model for prevention of addiction. *Journal of Ardabil University of Medical Sciences*.

[38] Hitchcock J. E., Schubert P. E., Thomas S. A. (2003). *Community Health Nursing: Caring in Action*.

[39] Morowatisharifabad M., Fadaeevash N., Allahverdipour H., Fallahzadeh H. (2012). *Study of Smoking Predictors Based on Prototype/Willingness Model Omong High School Students in Maragheh*.

[40] Li X., Mao R., Stanton B., Zhao Q. (2010). Parental, behavioral, and psychological factors associated with cigarette smoking among secondary school students in Nanjing, China. *Journal of Child and Family Studies*.

[41] Hemchayat M. (2003). *Predictors of Thai Adolescent Cigarette Smoking According to the Theory of Planned Behavior*.

[42] Krohn M. D., Skinner W. F., Massey J. L., Akers R. L. (1985). Social learning theory and adolescent cigarette smoking: a longitudinal study. *Social Problems*.

[43] Nofziger S., Lee H.-R. (2006). Differential associations and daily smoking of adolescents: the importance of same-sex models. *Youth & Society*.

[44] Hawkins J. D., Weis J. G. (2017). *The Social Development Model: An Integrated Approach to Delinquency Prevention. Developmental and Life-Course Criminological Theories*.

[45] Glanz K., Rimer B. K., Viswanath K. (2008). *Health Behavior and Health Education: Theory, Research, and Practice*.

[46] Ghasemi M., Sabzmakan L. (2015). Experiences of high school students about the predictors of tobacco use: a directed qualitative content analysis. *Journal of Education and Community Health*.

[47] Barati M., Niknami S., Hidarnia A., Allahverdipour H. (2014). Predictors of tobacco smoking in male adolescents in Hamadan based on the theory of planned behavior. *Journal of Education and Community Health*.

[48] Didarloo A., Sharafkhani N., Rezapour B., Moghaddam-Tabrizi F. (2022). *Predictors of Smoking Preventive Behavior Based on Empowerment Components Among Male Students of High Schools: A Cross-Sectional Study in Iran*.

